The article "Study of Inflammatory and Infection Markers in Periprosthetic Fluid: Correlation with Blood Analysis in Retrospective and Prospective Studies" was published in 2021. Journal: Biomed Res Int.

# Study of Inflammatory and Infection Markers in Periprosthetic Fluid: Correlation with Blood Analysis in Retrospective and Prospective Studies

**DOI:** 10.1155/2021/6650846

**Published:** 2021-03-19

**Authors:** Andrea Lisa, Cristina Belgiovine, Luca Maione, Andrea Rimondo, Andrea Battistini, Benedetta Agnelli, Matteo Murolo, Leonardo Galtelli, Marta Monari, Marco Klinger, Valeriano Vinci

**Affiliations:** ^1^Humanitas Clinical and Research Center-IRCCS, Via Manzoni 56, 20089 Rozzano Milan, Italy; ^2^Scuola di Specializzazione in Microbiologia e Virologia, Università degli Studi di Pavia, 27100 Pavia, Italy; ^3^University of Milan, Reconstructive and Aesthetic Plastic Surgery School-Clinica San Carlo-Plastic Surgery Unit-Paderno Dugnano (Milan), Italy; ^4^Humanitas University Department of Biomedical Sciences, Via Rita Levi Montalcini 4, 20090 Pieve Emanuele, Milan, Italy; ^5^Clinical Investigation Laboratory, Humanitas Clinical and Research Center, Via Alessandro Manzoni 56 20089 Rozzano Milano, Italy; ^6^Plastic Surgery Unit, Department of Medical Biotechnology and Translational Medicine BIOMETRA, Humanitas Clinical and Research Hospital, Reconstructive and Aesthetic Plastic Surgery School, University of Milan, Via Manzoni 56, Rozzano, Milan 20090, Italy

## Abstract

**Background:**

Surgical site infection represents the most severe complication in prosthetic breast reconstruction. Risk profiling represents a useful tool for both clinicians and patients.

**Materials and Methods:**

In our hospital, 534 breast reconstructions with tissue expander implants, in 500 patients, were performed. Several clinical variables were collected. In our study, we evaluated the different inflammatory markers present in the periprosthetic fluid and we compared them with the ones present in plasma.

**Results:**

The surgical site infection rate resulted to be 10.5%, and reconstruction failed in 4.5% of the cases. The hazard ratio for complications was 2.3 in women over 60 (CI: 1.3-4.07; *p* = 0.004), 2.57 in patients with expander volume ≥ 500 cc (CI: 1.51-4.38; *p* < 0.001), 2.14 in patients submitted to previous radiotherapy (CI: 1.05-4.36; *p* < 0.037), and 1.05 in prolonged drain use (CI: 1.03-1.07; *p* < 0.001). 25-OH, PCT, and total protein were less concentrated, and ferritin and LDH were more concentrated in the periprosthetic fluid than in plasma (*p* < 0.001). CRP (*p* = 0.190) and *β*-2 microglobulin (*p* = 0.344) did not change in the two fluids analyzed. PCT initial value is higher in patients who underwent radiotherapy, and it could be related to the higher rate of their postoperative complications. Patients with a tissue expander with a volume ≥ 500 cc show an increasing trend for CRP in time (*p* = 0.009).

**Conclusions:**

Several risk factors (prolonged time of drains, age older than 60 years, and radiotherapy) have been confirmed by our study. The study of markers in the periprosthetic fluid with respect to their study in plasma could point toward earlier infection detection and support early management.

## 1. Introduction

Breast cancer is the most common cancer among women worldwide [1], and it represents around 29% of all cancers in Italian women [2, 3]. The progressive increase in the diagnosis of breast cancer determines a simultaneous increase in the rate of postmastectomy breast reconstructions. For both simplicity and lack of donor site morbidity, prosthetic reconstruction is commonly adopted. Moreover, compared with autologous breast reconstruction, it presents shorter surgical time, decreased hospitalization, and quicker recovery [4, 5].

However, this surgery is not risk-free; early or late infections, wound dehiscence, or mastectomy skin flap necrosis may present. The most severe is surgical site infection which can lead to reconstructive failure and, in the worst cases, removal of the implant [6]. Infection rates following prosthetic breast reconstruction are reported. The latter are linked to several risk factors like previous chemotherapy and/or radiotherapy, smoking, higher BMI, larger breast size, and lymph node dissection [7–10], ranging from 1 to 35% [11, 12]. At the moment, no biochemical marker is able to provide an early detection of the local inflammatory state and to predict the risk of early or late postsurgical complications.

The periprosthetic fluid, which accumulates in the drains, is a waste fluid easily collected. It should be considered both a mirror of the processes occurring inside the pocket during the early postoperative period and a potential cause of local inflammation, being a direct connection with the external environment.

A longer time to drain removal is associated with an increased rate of infection [13], although little is known about drainage fluid: its origin, its biochemical composition, and its differences in patients with a regular postoperative course and in patients presenting complications. Either this fluid could derive from blood filtration or it may be a wound exudate that develops in the inflammatory phase of wound healing [14].

For the aforementioned reasons, we performed a retrospective study of 500 patients (534 prosthetic reconstruction) to analyze risk factors for infection. Moreover, we prospectively analyze drainage fluid to characterize it from a biochemical point of view.

## 2. Methods

### 2.1. Patient Selection

We conducted a retrospective analysis, IRB-approved, on patients who underwent unilateral/bilateral immediate postmastectomy tissue expander breast reconstruction at Humanitas Research Hospital from January 2013 to December 2016. Moreover, we performed a prospective analysis on 32 patients who underwent mastectomy and one-stage breast reconstruction at Humanitas Research Hospital between November 2016 and May 2017.

Demographic, reconstructive, and complication data were obtained from medical records and collected into a clinical database.

“Smokers” were defined as patients who continued to smoke throughout the perioperative period and/or those who stopped less than 4 weeks preoperatively. “Ex-smokers” are defined as patients who had stopped smoking between 1 and 12 months preoperatively. We have considered both groups as a single group since it has been observed that complication rates are similar in these two populations [10]. Patients were considered to have undergone neoadjuvant chemotherapy if they completed therapy within 6 weeks from mastectomy and subsequent reconstruction.

Surgical technique (total, nipple-sparing, and skin-sparing mastectomy), operative time, sentinel lymph node biopsy with or without axillary dissection, and expander brand and volume were also collected.

Infection was clinically defined considering the following signs or symptoms: fever (>38°), localized erythema, swelling, pain, wound dehiscence, expander exposure, and purulent drainage from deep incisions.

The cutoff between early and late infections was considered to be 30 days.

### 2.2. Surgical Technique

We performed first-stage breast reconstruction with a tissue expander or single-stage breast reconstruction with a definitive prosthesis, depending on breast characteristics, mastectomy type, intraoperative conditions, tissues' quality, and indication for subsequent radiotherapy. Closed drainage suction systems were placed in the subcutaneous tissue, in the periprosthetic pocket and, if axillary lymph node dissection was performed, also in the axilla. All tissue expander reconstructions were performed using anatomic and textured expanders with an integrated expansion port from either Mentor (Mentor Corporation, Santa Barbara, Calif.) or Allergan (Allergan Corporation, Marlow International, Parkway, Marlow, Bucks, SL7 1 YL, United Kingdom). No acellular dermal matrix (ADM) has ever been employed in the selected patients. Expanders were placed in a complete submuscular position and filled intraoperatively with a variable amount of saline. A reduced filling volume is indicated in smokers and patients submitted to previous radiotherapy (never more than 10% of overall volume). At complete wound healing, saline instillations started in the outpatient setting, and then, they were performed every two weeks. If radiotherapy was required for oncological reasons, expansions were interrupted and restarted 2-3 months after the last session of radiotherapy, according to skin conditions. The duration of hospitalization was around 1-3 nights. The compressive dressing placed after surgery was removed at the first consultation in the outpatient setting. Antibiotic prophylaxis consisted of cefazolin 2 g i.v. Intraoperatively, all patients received intravenous antibiotics, prolonged orally (cefazolin 1 g once a day) in the postoperative period until drain removal. Acetaminophen was prescribed as an analgesic therapy.

### 2.3. Postoperative Procedure and Periprosthetic Fluid Collection

The first consultation was planned 5 days postoperatively. The second consultation was planned about a week after. The following consultations were planned every week for the first month and then every 2-3 weeks, unless complications occurred. The drainage tubes were removed when the drained fluid was steadily less than 50 mL per day for a 3-day period. Whenever possible, fluid was collected from the drainage system into an EDTA and a serum test tube on the 1st postoperative day and at following outpatient consultations, and it was sent to the laboratory. Only patients from whom the drainage fluid was collected on the 1st postoperative day and at least another time (first or second outpatient consultations) were included in the study. The timing of the drainage collection is shown in Table 1.

### 2.4. Measure of Biological Markers

We analyzed the following parameters, considering their wide availability in the clinical routine as inflammatory markers and their moderate cost: 25-hydroxyvitamin D (25-OH), procalcitonin (PCT), ferritin, total protein, lactate dehydrogenase (LDH), C-reactive protein (CRP), and *β*-2 microglobulin. 25-OH was analyzed using the LIASON® 25 OH Vitamin D Assay, which is a direct and competitive immunological test, resting on the Chemiluminescence Immunoassay based on recombinant VlsE (CLIA) principle. The LIASON® BRAHMS PCT® II GEN test takes advantage of the CLIA principle in order to quantify PCT. ARCHITECT Ferritin is the Chemiluminescent Microparticle Immunoassay (CMIA) applied for the analysis of ferritin. Total protein was quantified through the ARCHITECT cSystems. The ARCHITECT Lactate Dehydrogenase 2P56 kit was applied to determine the dosage of LDH. ARCHITECT cSystems MULTIGENT CRP16 was used for the quantitative immunoturbidimetric determination of CRP. *β*-2 microglobulin was analyzed through the Abbott ARCHITECT cSystems.

### 2.5. Statistical Analysis

For the retrospective analysis, we used a proportional hazard Cox regression analysis. Factors with a significance level at univariable analysis under 0.1 were then submitted to a multivariable Cox regression analysis. Among the patients who had developed infection, the presence of possible risk factors for the explant was evaluated through logistic regression analysis. A *p* value less than 0.05 was considered significant. The analysis was carried out with Stata 13. For the prospective analysis, we explored different methods: Mann-Whitney test and paired *t*-test, and we performed a multivariable analysis. Statistical significance was set at *p* = 0.05. Chi-square or Fisher's exact test was used when indicated. Statistical analysis was performed with SPSS software (version 21.0; IBM Corporation, Armonk, NY).

## 3. Results

### 3.1. Risk Factors for Breast Reconstruction Failure: Retrospective Study

Over the 3-year study period, 534 consecutive tissue expander reconstructions were performed in 500 patients (Table 2). The overall surgical site infection (SSI) rate was 10.49% (56 out of 534, 95% CI: 8.02%–13.40%) among which 55.36% were early infection (31 out of 56) while 44.64% occurred after 30 days from the operation (late infections). Reconstructive failure, defined as expander removal, occurred in 24 patients (4.49% of the total sample and 42.86% of those who developed SSI). Reconstruction failure was determined by late infections in 54.17% of cases (13 patients out of 24).

In order to identify infection risk factors, we performed a univariable and multivariable statistical analysis (results in Table 3). Univariable analysis was also performed to identify risk factors for reconstructive failure in the group of patients who developed SSI, although we did not identify any risk factor (Table 4).

### 3.2. Prospective Study: Cohort Description

The main characteristics of the 32 patients are presented in Table 5.

### 3.3. Biological Marker of Infection: Plasma versus Periprosthetic Fluid

A preliminary analysis was performed comparing the fluids collected from the first patients using both EDTA and serum test tubes, showing that, on 77 parameter trends considered, 9 (12%) differences were recorded. Among the latter, 5 and 4 cases showed increasing trends with serum and with the EDTA test tube, respectively. Six differences were recorded in LDH, two in 25-OH, and one in *β*-2 microglobulin. All the remaining analyses were performed only using serum test tubes.

Time 0 collection was analyzed in order to investigate the range of variability of the parameters and therefore the cutoff that we used to define the stability of each parameter in time. The results are presented in Table 6.

The comparison of the distribution of the parameters between the periprosthetic fluid and the referred reference interval in plasma is presented in Table 7 (chi-square or Fisher's exact test was used when indicated). The only variables whose distributions did not differ from the plasmatic ones were CRP (*p* = 0.190) and *β*-2 microglobulin (*p* = 0.344). 25-OH, PCT, and total protein were less concentrated in the periprosthetic fluid than in plasma (*p* < 0.001), whereas ferritin and LDH were more concentrated in the periprosthetic fluid than in plasma (*p* < 0.001).

The distributions of PCT and CRP in periprosthetic fluid and plasma are shown in Figure 1.

### 3.4. CRP as a Marker of Early Infection

We categorized the trends for each parameter during fluid collection (between the last and the first), and they are reported in Table 8. 25-OH showed a stable trend in 25 (78%) patients, with only 6 (19%) patients presenting increasing values in time. PCT was stable in 15 (47%), decreasing in 7 (22%), and increasing in 10 (31%) patients. Ferritin was higher at the last collection with respect to the first one in 20 patients (63%) and stable in 11 patients (34%). LDH tended to decrease in 24 patients (75%) and remained constant in 8 patients (25%). Total protein was stable in 28 (88%) patients, with only 4 (13%) showing a decreasing trend. CRP was stable in 17 (53%), decreasing in 5 (16%), and increasing in 10 (31%) patients. Eventually, most patients (94%) had an increasing trend of *β*-2 microglobulin in time.

We focused our attention on CRP. CRP is the only parameter that is concentrated in a similar manner in blood as well as in drainage fluid and analyzable trends. Also, *β*-2 microglobulin has shown a similar distribution in plasma and in periprosthetic fluid; however, 94% of patients had an increasing trend; therefore, it could not be investigated. We analyzed the correlations between patients and surgery characteristics and an increasing trend for CRP in time in the periprosthetic fluid. Patients with a tissue expander with a volume ≥ 500 cc had a higher probability of showing an increasing trend for CRP in time (OR = 21.600, 95%CI = 2.135-218.579, *p* = 0.009), and this was the only factor which tested statistically significant in univariate analysis (Table 9). Patients with a BMI > 23 showed an increasing trend of CRP in time (OR = 4.083, 95%CI = 0.818-20.376, *p* = 0.086).

## 4. Discussion

Breast reconstruction has been shown to improve postmastectomy quality of life, to aid in coping with the diagnosis of breast cancer, and to decrease psychologic morbidity [10, 15, 16]. Tissue expander/prosthesis reconstruction is a well-established technique which can provide excellent aesthetic results although surgical site infection still represents the highest predictive factor of subsequent implant failure [17].

A successful reconstruction starts with careful patient selection and meticulous preoperative planning. Several studies have attempted to identify risk factors for complications following prosthetic breast reconstruction [6–12].

Our study firstly provides data about 534 consecutive tissue expander/implant reconstructions in 500 women evaluating the impact of clinical risk factors on the development of local infection. Secondly, we conducted a preliminary prospective analysis of 32 patients who underwent mastectomy and implant-based breast reconstructive surgery aimed at investigating the microenvironment of the fluid collected in the periprosthetic pocket drainage system.

Previous studies about this topic reported different features as markers of early detection of infection leading to possible implant loss: obesity [18–22], smoking [17–19, 22], hypertension [17, 19], chemotherapy [23] and radiotherapy [24], age [17, 19, 23], drainage maintenance [13], and also volume of the tissue expander [18].

In our work, the main predictive factor is represented by expander volume. This variable is directly related to breast volume since we select it according to the patient's anatomic features. We are convinced that the main cause of local infection in these patients is related to delayed seroma. The latter may be determined either by increased fluid in the periprosthetic space, which indeed appears to be greater in these patients, or by a reduced vascularization of the mastectomy flap in bigger breasts. This data is confirmed also by the prospective analysis in which we found that patients with a tissue expander with a volume ≥ 500 cc had a higher probability of showing an increasing trend for CRP in time (*p* = 0.009). Breast weight represents an interesting variable to consider together with expander volume. Actually, this parameter is missing in our clinical database, but we will introduce it in future research.

It has been demonstrated, also in previously published reports, that the administration of neoadjuvant or adjuvant chemotherapy does not affect the risk of complications. On the other hand, radiotherapy needs a more complex analysis. Indeed, we found that a history of irradiation increases the risk for the development of local infection. Our group does not consider this condition as a relative adverse indication for tissue expander/implant reconstruction [25]. Indeed, if we observe the OR of reconstruction failure previous radiation, it appears to be inferior to 1, although without statistical significance. In our opinion, this observation is due to the fact that previously irradiated patients are more strictly evaluated for the known risk of local infection and in a certain amount of patients we actually consider local infection as redness related to previous radiodamage. Moreover, these patients, analyzed in the prospective study, showed an increased probability of having a higher initial value of PCT (*p* = 0.033).

Interestingly, as already observed by Power et al. [13], we detected a statistically significant correlation between time of drainage maintenance and development of local infections. In particular, if we set a cutoff of 21 days, we observed a statistical significant increase in local infections. As already declared, it is possible that prolonged fluid production determines a delayed healing and that the drains could act as a direct conduit from the external environment into the periprosthetic space.

For this reason, we agree that for a period of drainage maintenance greater than 3 weeks, the risk of maintaining the drain outweighs the risk of fluid collection.

The main aim of our small cohort of prospective analysis was to investigate the composition of the periprosthetic fluid in order to elucidate the possible role of the different inflammatory parameters both in the process of capsule formation and in the risk of development of postoperative complications. First of all, analyzing inflammatory markers, we found that the microenvironment of the periprosthetic fluid presents a different composition with respect to plasma. This could mean that not only is the periprosthetic fluid composed of extravasated blood but also it could represent a particular microenvironment in which inflammatory processes occur immediately after surgery, since the differences with plasma were evident since the first postoperative day. In particular, 25-OH, PCT, and total protein were less concentrated in the periprosthetic fluid than in plasma, whereas ferritin and LDH were more concentrated in the periprosthetic fluid (*p* < 0.001). The only parameters whose distribution did not differ from the plasmatic ones were CRP (*p* = 0.190) and *β*-2 microglobulin (*p* = 0.344).

These data could allow an improvement in our clinical practice: on the one hand, this work represents one of the largest single-center European report, and on the other hand, from the analysis of our results, we aim to obtain valuable information on the association between clinical variables and outcomes in our specific population.

Furthermore, our preliminary study showed that the composition of drainage microenvironment following mastectomy and implant-based breast reconstruction is different from the plasmatic one in terms of inflammatory parameters. This data suggests that the fluid could represent the expression of a complex local inflammatory process. Moreover, the values of PCT and CRP in the periprosthetic fluid, found, respectively, in patients who had undergone previous radiotherapy and patients with a tissue expander with a volume ≥ 500 cc, could be potentially related to a higher risk of developing infectious complications. These findings could allow us to identify value cutoffs for inflammatory parameters at specified postsurgical times able to predict an increased risk for postoperative complications, and they could allow a better tailoring of the postoperative antibiotic prophylaxis, as specific subsets of patients could be addressed to a more aggressive prophylaxis, whenever risk factors for infection were recognized based on the periprosthetic fluid collection during the first outpatient consultation. Further studies are needed in order to confirm the preliminary results and to better investigate the periprosthetic microenvironment, including other inflammatory parameters such as TNF-*α*, IL-1, IL-6, TGF-*β*, and pentraxin with special attention to potential correlations with the clinical outcomes. Another point to strengthen our analysis is suggested by Stewart et al. who performed the count of neutrophils present in the periprosthetic space to discover infections [25]. Moreover, a larger sample of patients should be included, in order to analyze possible correlations between the composition of the fluid and the clinical outcomes of the reconstructions, which could be possible only when a sufficient number of infectious complications will be recorded, considering their relatively low incidence rate.

## Figures and Tables

**Figure 1:** (a) PCT is less concentrated in the periprosthetic fluid than in plasma (*p* < 0.001). (b) CRP shows a similar distribution between periprosthetic fluid and plasma (*p* = 0.190).

**Table 1:** Timing of fluid collection.

Time	No. of patients	Median range (days)
0	32	1 (1-1)
1	28	5 (5-10)
2	25	12 (9-20)

**Table 2:** Sample characteristics.

	All
*N*	534
Age (years)	51 ± 10
Age (>60 years)	88 (16.48%)
BMI	24.3 ± 4.4
BMI (>30)	51 (9.57%)
Smoke (actual + ex)	154 (28.84%)
Diabetes	15 (2.81%)
Autoimmune pathologies	34 (6.37%)
Chemotherapy	290 (54.31%)
Previous RT	46 (8.61%)
RT	181 (33.90%)
Expander brand (Mentor)	146 (27.34%)
Expander volume (>500 mL)	117 (21.91%)
Axillary dissection	252 (47.19%)
Bilateral	36 (6.74%)
RMI	62.2 ± 21.5
Total duration	149.2 ± 55.4
Time of drainage (days)	19.6 ± 7.8

**Table 3:** Hazard ratios for risk factors.

	Univariable	*p*	Multivariable	*p*
	HR (95% CI)		HR (95% CI)	
Age	1.04 (1.02–1.06)	0.001	1.03 (1.00-1.06)	0.032
Age (>60 years)	2.30 (1.30–4.07)	0.004		
BMI	1.04 (0.98–1.09)	0.183		
BMI (>30)	1.60 (0.76–3.38)	0.220		
Smoke (active + ex)	1.37 (0.79–2.36)	0.261		
Diabetes	1.31 (0.32–5.35)	0.712		
Autoimmune pathologies	1.49 (0.60–3.74)	0.394		
Chemotherapy	0.77 (0.46–1.31)	0.337		
Neoadjuvant chemotherapy	0.37 (0.12–1.18)	0.092		
Adjuvant chemotherapy	1.02 (0.60–1.72)	0.954		
Previous RT	2.14 (1.05–4.36)	0.037	—	0.068
Expander brand (Mentor)	1.17 (0.66–2.07)	0.582		
Expander volume (>500 mL)	2.57 (1.51–4.38)	0.001	2.02 (1.12–3.65)	0.019
Axillary dissection	0.83 (0.49–1.41)	0.486		
Bilateral	0.80 (0.25–2.56)	0.708		
Mstec (×10 minutes)	0.99 (0.93–1.06)	0.854		
RMI	0.99 (0.98–1.01)	0.283		
Total duration (×10 minutes)	0.99 (0.94–1.04)	0.647		
Time of drainage (days)	1.05 (1.03–1.07)	<0.001	1.03 (1.01–1.06)	0.014

**Table 4:** Risk factors for reconstruction failure in SSI patients.

	Reconstruction failure		*p*	OR (95% CI)	*p*
	Yes	No			
*N*	24	32			
Age (years)	54 ± 12	56 ± 12	0.481	0.99 (0.95–1.03)	0.619
Age (>60 years)	8 (33.33%)	9 (28.13%)	0.772	1.28 (0.41–4.02)	0.675
BMI	25.6 ± 4.7	24.7 ± 5.2	0.230	1.04 (0.93–1.15)	0.527
BMI (>30)	4 (16.67%)	4 (12.90%)	0.718	1.35 (0.30–6.06)	0.695
Smoke (actual + ex)	12 (50.00%)	8 (25.00%)	0.090	3.00 (0.97–9.30)	0.057
Diabetes	2 (8.33%)	0	0.179	1	
Autoimmune pathologies	3 (12.50%)	2 (6.25%)	0.642	2.14 (0.33–13.96)	0.425
Chemotherapy	11 (45.83%)	16 (50.00%)	0.793	0.85 (0.29–2.44)	0.758
Neoadjuvant chemotherapy	0	3 (9.38%)	0.252	1	
Adjuvant chemotherapy	11 (45.83%)	13 (40.63%)	0.788	1.24 (0.42–3.60)	0.697
Previous RT	2 (8.33%)	7 (21.88%)	0.274	0.32 (0.06–1.73)	0.187
RT	5 (20.83%)	8 (25.00%)	0.760	0.79 (0.22–2.81)	0.715
Expander brand (Mentor)	9 (37.50%)	8 (25.00%)	0.384	1.80 (0.57–5.69)	0.317
Expander volume (>500 mL)	11 (45.83%)	12 (37.50%)	0.590	1.41 (0.48–4.13)	0.531
Axillary dissection	11 (45.83%)	13 (40.63%)	0.788	1.24 (0.42–3.60)	0.697
Bilateral	2 (8.33%)	1 (3.13%)	0.571	2.82 (0.24–33.05)	0.409
Mstec (×10)	9.81 ± 3.80	7.93 ± 3.10	0.091	1.18 (0.99–1.42)	0.071
RMI	58.2 ± 19.8	59.8 ± 13.9	0.481	0.99 (0.96–1.03)	0.716
Total duration (×10)	15.63 ± 5.19	13.92 ± 3.07	0.344	1.12 (0.96–1.30)	0.158

**Table 5:** Patients' characteristics.

Characteristics	*n* = 32
Bilateral intervention	3 (9%)
Median age (range)	52 (32-69)
Median BMI (range)	22.9 (17.4-33.4)
Current smoker	9 (28%)
Previous breast surgery	11 (34%)
Previous RT	8 (25%)
Previous CT	5 (16%)
Prophylactic mastectomy	4 (13%)
Demolitive surgery	
Radical mastectomy	10 (31%)
Nipple-sparing mastectomy	19 (59%)
Skin-sparing mastectomy	3 (9%)
Implant type	
Expander	27 (84%)
Immediate prosthesis	5 (16%)
Median implant size (cc) (range)	400 (125-650)
Median prefilling expander volume (cc) (range)	100 (20-400)
Operated side	
Bilateral	3 (9%)
Right	14 (44%)
Left	15 (47%)
Contralateral intervention	2 (6%)
Axillary dissection	6 (19%)

**Table 6:** Range of variability of the parameters and cutoff for stability adopted.

Parameter	Unit	Min	Max	Ratio max/min	Cutoff for stability
25-OH	ng/mL	<4.0	39.5	10	1/2 or ×2
PCT	ng/mL	<0.02	3.71	185	1/3 or ×3
Ferritin	ng/mL	71	2910	41	1/3 or ×3
LDH	IU/L	974	>6650	7	1/2 or ×2
Total protein	g/L	20.3	85.7	4	1/2 or ×2
CRP	mg/dL	0.03	1.10	37	1/3 or ×3
*β*-2 microglobulin	mg/L	<0.25	2.93	12	1/2 or ×2

**Table 7:** The comparison of the distribution of the parameters between the periprosthetic fluid and the plasmatic referred reference interval (chi-square or Fisher's exact test was used when indicated).

Parameter	Unit	Plasmatic reference interval	Median value in fluid	Fluid values < min plasma	Fluid values > max plasma	*p* value
25-OH	ng/mL	30.0-100.0	18.5	26 (81%)	/	<0.001
PCT	ng/mL	0.00-0.50	0.04	/	3 (9%)	<0.001
Ferritin	ng/mL	20-250	346	/	22 (69%)	<0.001
LDH	IU/L	125-243	3791	/	32 (100%)	<0.001
Total protein	g/L	60.0-80.0	46.3	26 (81%)	1 (3%)	<0.001
CRP	mg/dL	0.01-0.50	0.17	/	4 (13%)	0.190
*β*-2 microglobulin	mg/L	0.97-2.64	1.60	/	1 (3%)	0.344

**Table 8:** All trends for the 32 patients analyzed for each parameter (chi-square or Fisher's exact test was used when indicated).

Parameter	Stable trend	Decreasing trend		Increasing trend	
	*n* (%)	*n* (%)	*p* value	*n* (%)	*p* value
25-OH	25 (78%)	1 (3%)	N.A.	6 (19%)	0.004
PCT	15 (47%)	7 (22%)	0.237	10 (31%)	0.022
Ferritin	11 (34%)	1 (3%)	N.A.	20 (63%)	<0.001
LDH	8 (25%)	24 (75%)	<0.001	/	N.A.
Total protein	28 (88%)	4 (13%)	0.043	/	N.A.
CRP	17 (53%)	5 (16%)	0.063	10 (31%)	0.005
*β*-2 microglobulin	2 (6%)	/	N.A.	30 (94%)	<0.001

**Table 9:** Univariate analysis for the CRP increasing trend.

Covariates	CRP increasing trend (10/32 = 31%)			
	*n* (%)	OR	95% CI	*p* value
Bilateral surgery Unilateral surgery	1/3 (33%) 9/29 (31%)	1.111	0.089-13-894	0.935
Age > 52 yr Age ≤ 52 yr	6/19 (32%) 4/13 (31%)	1.038	0.226-4.768	0.961
BMI > 23 BMI ≤ 23	7/15 (47%) 3/17 (18%)	4.083	0.818-20.376	0.086^∗^
Smoker Nonsmoker	4/9 (44%) 6/23 (26%)	2.267	0.453-11.349	0.319
Prophylactic indication Therapeutic indication	1/4 (25%) 9/28 (32%)	0.704	0.064-7.742	0.774
Total mastectomy Nipple-skin-sparing mastectomy	5/10 (50%) 5/22 (23%)	3.400	0.693-16.687	0.132
Immediate prosthesis Expander	0/5 (0%) 10/27 (37%)			0.155
Expander ≥ 500 cc Expander < 500 cc	9/14 (64%) 1/13 (8%)	21.600	2.135-218.579	0.009^∗^
Prefilling volume > 100 cc Prefilling volume ≤ 100 cc	4/10 (40%) 6/17 (35%)	1.222	0.244-6.111	0.807
Contralateral intervention No contralateral intervention	1/2 (50%) 9/30 (30%)	2.333	0.131-41.554	0.564
Axillary dissection No axillary dissection	3/6 (50%) 7/26 (27%)	2.714	0.440-16.750	0.282
Previous surgery No previous surgery	3/11 (27%) 7/21 (33%)	0.750	0.150-3.742	0.726
Chemotherapy No chemotherapy	2/5 (40%) 8/27 (30%)	1.583	0.221-11.361	0.648
Radiotherapy No radiotherapy	3/8 (38%) 7/24 (29%)	1.457	0.271-7.821	0.661
Subcutaneous drainage removal > 6 days Subcutaneous drainage removal ≤ 6 days	3/13 (23%) 6/18 (33%)	0.600	0.119-3.032	0.537
Pocket drainage removal > 18 days Pocket drainage removal ≤ 18 days	5/14 (36%) 5/17 (29%)	1.333	0.294-6.043	0.709

^∗^Variables with a *p* value < 0.1 entered the multivariate model.

## Data Availability

Data are available on request.
